# The Study of Immersive Physiology Courses Based on Intelligent Network through Virtual Reality Technology in the Context of 5G

**DOI:** 10.1155/2022/6234883

**Published:** 2022-05-14

**Authors:** Ling Ma, Wei Zhang, ManJin Lv, JingNing Li

**Affiliations:** Higher Vocational Supervision Office, Yongzhou Vocational and Technical College, Yongzhou 425000, Hunan, China

## Abstract

The current boom in Internet technology has paved the way for the research and evolution of various technologies related to it. One such technology is immersive virtual reality (IVR). Immersive technology is referred to as creating a reality-like experience by combining the physical world with digital reality. There are two main types of immersive technologies. Immersion in virtual reality is the perception of being physically present in an artificially created world. Perception is artificially created by images, videos, sounds, or other stimuli with the help of a virtual reality (VR) system that the user is connected to. VR uses rendered computer-generated simulations and results in a complete sense of immersion. Immersive virtual reality (immersive VR) refers to engaging users in an artificial environment that replaces their natural surroundings and fully engages them with the artificially created environment. In this research, we will research immersive physiology courses based on artificial intelligence combined with wireless network VR technology in the context of 5G. The teaching methodology has been kept up-to-date along with the technology. Teaching physiology courses also incorporate new technologies like immersive technologies. The use of technology in anatomy and physiology courses allows students to view structures and physiological concepts in a realistic environment. Virtual dissection in 3D is available with a life-like artificial environment. Students can attend the classes with VR headsets, laptops, or smartphones to experience immersive and interactive 3D classes. This advanced technology enhances and empowers the students to learn from real-life situations like those available in the classes. In this research, CNN with AI is proposed for effective learning of physiology courses. This algorithm is compared with the existing NNGA, KNN, and Random Forest, and it is observed that the proposed model has obtained an accuracy of 99%.

## 1. Introduction

There is a lot of promise in virtual reality (VR), just like with smartphones and the Internet. Head-mounted displays and handheld controllers are used in virtual reality (VR) to make computers more intuitive and natural to use. New forms of global communication are possible, but with a human touch that has never been seen before. If they are standing together or face-to-face, it is practically hard to distinguish which is which. According to estimates, virtual reality will be used on a regular basis by the vast majority of Internet users all over the world in the next several years [1]. Virtual reality is expected to have a big impact on the future of mobile networks, particularly 5G networks (VR). However, there is a slew of technical obstacles that must be addressed before it can be widely used. Cutting-edge solutions and fundamental research from a variety of fields are necessitated by VR's high throughput, low latency, and dependable connectivity requirements [2]. Immersive VR's success hinges on overcoming a slew of issues across several fields of study. As a 5G use case, the researcher highlighted the necessity of VR technology (and beyond). While studying three virtual reality (VR) cases, the author also offered numerical results under a variety of storage, computation, and network configurations [3]. Virtual reality research is still missing in practice, despite the many hypotheses that have been put forth and the reasons why the public should take the lead. By using recessed rendering, the author believes that wide-field displays can be rendered faster by reducing visual detail in areas that are not directly in the path of an eye's movement [4]. By conducting a user survey, the researcher discovered that people's impressions of their peripheral vision when viewing today's displays may be improved. A discernible target picture was created to develop and produce a centralized renderer after these insights were verified on desktops and head-mounted displays using high-speed gaze tracking [5]. Despite the fact that researchers created a useful recessed rendering technique, people never tested it. People think virtual reality (VR) dispersion therapies can be used to successfully alleviate pain [6]. A multimodal pain sequence (alternating thermal stimulation and distal stimulation) was administered to 74 healthy participants over the course of 18 minutes (average age: 29 years, 37 women). Subjective pain intensity and enjoyment scales of 0–10 points and a nine-point scale, respectively, were used to assess the subjects' subjective pain and enjoyment [7]. In this study, researchers discovered that virtual reality diversions, such as immersive virtual reality, can help people cope with pain. According to the researcher, virtual reality (VR) and computer-generated interactive environments (CII) can assist people in better understanding the issues they face and learning how to overcome them [8]. It was a thorough investigation into the evidence that was available. There were a total of 285 research discoveries, with 86 of them being assessments, 45 being theoretical breakthroughs, and 154 being treatments. In this study, we discovered that exposure to virtual reality can help to lower anxiety, although, there are just a few effective studies and treatment alternatives at this time [9].

In order to create the virtual human's animation, it is necessary to interpolate the virtual human's centre of gravity and then render the model position gained in each frame obtained from the interpolation [10]. There are numerous video storage, playback, and freezing choices accessible when three-dimensional data on human motion is used to synthesize a virtual human animation [11]. Additionally, the system is capable of displaying and playing back film captured by a camera at the same time, allowing for an intuitive comparison of the athletes' moves [12]. A 3D virtual human body simulation video can be created using VC++6.0 as a development tool for coaches to edit the sports of extraordinary domestic and international athletes on the spot [13]. A camera is used to gather three-dimensional motion data, which is then transported to a three-dimensional virtual human model, where it can be utilized to recreate an athlete's technical activities [14]. In addition, subjectivity in the application of artificial intelligence technology has supplanted the conventional subjects and purposes of training (education robot and intelligent tutor system). However, this does not imply that instructors are no longer needed in today's society [15]. Traditional “teaching, preaching, and answering riddles” tasks for instructors have given way to “creating, advancing, assisting, and caring” ones. It is the instructor's responsibility to develop and implement learning activities, to encourage the educational process, and to provide psychological assistance to students who are experiencing psychological difficulties [16]. With today's technology, it is difficult to recreate something as spectacular as this.

Machine learning and deep learning and the use of artificial intelligence in traditional fields such as biology and information theory, are currently being studied in higher education institutes in my country [17]. The scientific research conducted in my nation is greatly impacted by what takes place in its universities. A bigger investment in artificial intelligence research and the development of students' scientific research conceptions and abilities is required in the current world environment [18]. You must first identify the “difficult activities” from the “initial motion portion” as a starting point for your investigation. It creates a 3D scene and a virtual human body model depending on the user's specifications. The system comes with a virtual character library [19]. A number of human body models can be selected by the technician or administrator based on the requirements of the user. Creating a virtual training environment that includes sports-related reference objects is necessary. Real-time recording of an individual's physical activity is taking place. Two cameras and a computer are typically involved in this process. Key frame images are manually extracted from video files captured during the simultaneous shooting method using the cameras' existing computer technology [20]. Motion data for a three-dimensional animation of the human body is calculated using two engraved two-dimensional motion data for each joint of the human body concurrently in order to extract the moving human body. Recreating what you've seen, this function's goal is to play the 3D body motion data at a defined frame rate and create an animation once it has been rendered in the 3D scene [21]. All of the students' motions are recorded by the computer. A high-quality simulation allows students to examine their activities from a number of angles and perspectives, improving their performance. Fundamentally, the simulation system needs to “reproduce activity.” This visible and intuitive instruction is provided to the students by the trainer, who can also demonstrate some still under-researched technical actions and watch the students' technical actions from various viewpoints [22]. Get the statistics on movement number four! Depending on the demands of coaches and trainers, the system may provide feedback on a wide range of athlete-related variables, including heart rate, blood pressure, and more. Better management of sports risk can be achieved while also reducing risk objectively. The trainees' performance metrics are monitored [23]. The training effect of the real-time picture presentation coaches are able to compare athletes' performances horizontally and vertically and comprehend their training process and training in time and whether there are positive changes in the outcomes after the conclusion, thanks to real-time charts of athletes' performance data. Re-examination of the data has taken place. Because of the high prevalence of errors and unpredictable causes, it is necessary for the system to smooth and remove noise from raw data in order to make it useable [24]. It is now possible to further improve and develop technology activities, such as integrating multiple technological operations into a single platform. In real time, two videos are compared. Because of the use of virtual reality technology in athletics, it is possible to improve training and competitiveness while maintaining or even lowering costs. Sports as a tool for preserving national health and well-being also benefit greatly from this. It is becoming increasingly important in today's field of sports training to study and use it [25]. There is no existing detailed study about the immersive physiology courses using machine learning. This study focused on an immersive physiology course based on artificial intelligence combined with wireless network virtual reality technology in the context of 5G.

The contribution of this study is as follows:

- This study offered a new approach to teacher quality in education courses at higher learning institution.
- The study proposed the convolution neural network with a wireless network, which can increase time saving.

### 1.1. Motivation of the Study

Physiology education will be seen as an important element of health education and a reflection of the school system. A physiology course teacher is in charge of giving students physiology education courses focused on AI and/or health teaching. Using student physiology courses, this study proposed a new method of teacher quality in education courses at higher education institutions. The framework presented by humans could indeed enhance the general broad validity of conventional wireless networks along with training time by combining conventional neural network algorithms with wireless network methods. Education is viewed as an important part of health education and is also a reflection of virtual reality technologies in the context of the 5G system. A physiology course teacher is in charge of giving students physiology education courses focused on AI and/or health teaching. Using student physiology courses, this study provided a new approach to teacher quality in education courses at institutes of higher learning. By combining convolution neural network algorithms with wireless network methods, the framework proposed by humans can increase the training time.

## 2. Materials and Methods

Immersive technology is an artificially intelligent technique that uses real-life, live-rendered computer-generated imagery, sound effects, etc., that seems to be more engaging to the user so that the user can perform physical activity as in reality by experiencing the artificially generated environment. Students, with the help of VR kits such as headsets, can experience this 3D dynamic view of a computer-generated artificial environment. The wireless network system and 5G technologies play a major role in this proposed model. In the field of telecommunications, 5G technology is of importance.

5G is referred to as the 5th generation mobile network, which is an updated wireless network communication model that aids in faster data transfer. 5G enables an easy network model that connects machines, objects, and devices virtually. 5G wireless technology is a reliable technology that delivers various applications to users. They are higher data speeds, lower latency, and improved network capacity and availability. Cellular phone companies have already deployed this technology to most of the current users of cell phones. In the case of physiological studies, students can use their cell phones along with the VR headset for their classes. The physiology courses deal more with human body-related and biochemistry-related studies. It is always necessary for the students to have a physical experience. More and more practise tests are involved in the traditional course structure. These are carried out in VR to engage the students and interactively educate them. Wireless Network Systems are those that provide wireless connectivity in any living environment, including homes, hospitals, educational institutions, and businesses. This technology uses various kinds of sensors to make things smarter. One such service is connectivity to the Internet, which is deployed in the proposed system. The data are shared with the institutions that provide the physiological courses seamlessly with the help of Internet technologies and the latest telecommunication technologies such as 5G. Certain studies, for example, physical dissection in anatomy, physical studies, bodily studies, biochemical studies, and so on. This provides the students with an interactive way of learning. VR technology also finds other applications in the field of physiological studies, such as physiotherapy. It is used to treat partially paralysed stroke patients with an interactive VR technique, thus leading to various improvements in their body activity. Thus, virtual reality technology is deployed in the physiological courses with the help of wireless 5G technologies, and promising results are obtained as a result of this research. This process is depicted in Figure 1. For performing the virtual reality, another technology named cloud computing is utilized to reduce the graphical hardware and computational resources that need to be installed in the local device. In this scenario, to provide higher integrity among the resources and to maintain the privacy of the nodes, Artificial Intelligent technology can be implemented.

The analysis indicators of the education physiological quality of education are *x*; the western surface nodes are *φ*_*i*_, as are the output nodes *i*, which appears to be the analysis value of physical quality education. Because the input image device broadcasts data directly to a frame node's centre, the output of the input layer node equals to the input; the output information of a midlayer base station makes significant contributions of an output node; and the activation function only has one base station, which also receives the input of a middle layer node and produces an output; the teaching standard evaluation effects.

Input data node *m*_*i*_, *i*={1,2,…, *x*}, where *x* represents the evaluation of teaching quality, the following equation represents the input to a *H* middle of a specimen node:

(1) $$\begin{array}{c} H_{j}=\sum_{j=1}^{x}\varphi_{ij}m_{i}. \end{array}$$

The results or information (course contents) obtained from the base station (server node at the university) to the node (student's system) are shown in the following equation:

(2) $$\begin{array}{c} R_{j}=\sum_{j=1}^{x}\frac{1}{{\left\{1+{\left[{\left(\sum_{i=1}^{x}\varphi_{j}R_{j}\right)}^{-1}-1\right]}^{2}\right\}}^{\prime }}=\sum_{j=1}^{x}\frac{1}{\left[{\left(H_{j}^{-1}-1\right)}^{2}\right]}, \end{array}$$

where *φ*_*j*_ denotes this same power from an information node's ground station *H*_*j*_^−1^ to such a frame node's centre *j* and *R*_*j*_ signifies the graph's factor and the *i*th teaching quality evaluation index.

Node of activation function: there are only *S* nodes in the output units (as shown in equation (3)), and the data are the high speed of the frame node's centre:

(3) $$\begin{array}{c} S=\sum_{j=1}^{x}\frac{1}{{\left\{1+{\left[{\left(\sum_{i=1}^{x}\varphi_{j}R_{j}\right)}^{-1}-1\right]}^{2}\right\}}^{2^{\prime }}}. \end{array}$$

The learning optimal control technique is defined as the mean score of such sum of the squares sum ∑_*i*=1_^*x*^*φ*_*j*_*R*_*j*_ of an error is between overall performance and the quantification value of *G* measurements and is displayed in the following equation:

(4) $$\begin{array}{c} G=\left(\frac{1}{M}\right)\sum_{m=1}^{x}{\left[\bar{s}-s\right]}^{2}=\left(\frac{1}{M}\right)\sum_{m=1}^{x}G_{j}. \end{array}$$

Despite the convolutional neural network evaluation processes changing *δG* framework, the goal of network teaching appears to be to minimize *τ* by modifying the network's authentication and authorization. The training algorithm technique *δc*_*ij*_ is used to adjust the delinking and is presented in the following equation:

(5) $$\begin{array}{c} G_{ij}=\sum \left\{\begin{array}{c} \varphi_{ij}=-\tau \left(\frac{\delta G}{\delta c_{ij}}\right),\\ \varphi_{j}=-\tau \left(\frac{\delta G}{\delta \varphi_{ij}}\right). \end{array}\right. \end{array}$$

Furthermore, for such a rate of learning, the *d*_*i*_*φ*_*j*_*R*_*j*_^2^ quantity of interaction optimizing parameters between the information data network and the medium surface access point is then shown in the following equation:

(6) $$\begin{array}{c} \varphi_{ij}=d_{i}\varphi_{j}R_{j}^{2}\left[1-\sum_{i=1}^{x}\varphi_{ij}d_{j}\right]\omega_{j}. \end{array}$$

The number of connection optimizing parameters is given in the following equation:

(7) $$\begin{array}{c} \varphi_{j}=\sum_{j=1}^{r}s^{2}R_{j}\left[1-\sum_{j=1}^{r}\varphi_{j}R_{j}\right]{\left[\bar{s}-s\right]}^{2}. \end{array}$$

So, to use this framework, the neural network's interaction weight can be defined using the ∑_*j*=1_^*r*^*φ*_*j*_*R*_*j*_ optimization technique of a specific neural network, and the inaccuracy across both overall performance and various sample values can be significantly lowered.

The system is in a higher optimization process, as shown in equation (8), by using an optimised neural network:

(8) $$\begin{array}{c} \min\left(G\right)=\sum_{j=1}^{r}\int \left(\varphi_{1},\ldots ,\varphi_{x}\right), \end{array}$$

where min(*G*) is as a whole inaccuracy of training phase and *φ*_1_,…, *φ*_*x*_ are the constant weights after strong united numbering, which include not only the weights of the network of input access to data points along with generally affecting endpoints but also the prediction models of centre node and output node modules, and *n* represents the number of system parameters. Among many of them, $\bar{s}$ and *s* are *φ*_1_ variables that represent the upper and lower limits of change.

The optimization algorithm is a low-capacity problem inside the process of analytical algorithms. Because an individual's area of interest is roughly equivalent to ∫(*φ*_1_,…, *φ*_*x*_) ability, the description of such an optimization problem has a massive effect on genetic algorithms. Because of the close navigation companionship between the *U* − *G* optimization process and the optimization method, the *G* < *U* strength training computational methods outlined are used in the following equation:

(9) $$\begin{array}{c} \int_{i}=\sum_{i=1}\left\{\begin{array}{cc} U-G & G<U,\\ 0 & G\geq U. \end{array}\right.\; \end{array}$$

Equation (9) represents the training optimization model, in which *G* represents the sum of all *G* ≥ *U* in the current generation. The recommendations below are used for *M*_*r*_ classification of genetic process parameters in order to accept responsibility for the ∫_1_(*U* − *G*)/*U* ∈ [0,0.5] efficiency of integration and to minimize unnecessary integration caused by efficient gene declassification of the following equation:

(10) $$\begin{array}{c} M_{r}=\left\{2\left(\frac{\int_{1}U-G\;G<U}{U}\right),\frac{\int_{1}\left(U-G\right)}{U}\in \left[0,0.5\right].\right. \end{array}$$

The min and max technique can be used for normalization handling ∫_1_(*U* − *G*)/*U* ∈ [0.5, 1] as it is an implementation for processing information that can effectively maintain its own original meaning while causing no data redundancy. The normalization equation to use for this document for these kind of input data are as follows:

(11) $$\begin{array}{c} M_{r}=\left[1-2\left(1-{\left(\frac{\int_{1}U-G\;G<U}{U}\right)}^{2}\right)\right],\frac{\int_{1}\left(U-G\right)}{U}\in \left[0.5,1\right]. \end{array}$$

The method of compressing a huge variety of information into the scope [0, 1] is known as standardization ∫_1_(*U* − *G*)/*U* ∈ [0.5, 1]. The solution to the standardization is represented in the following equation:

(12) $$\begin{array}{c} d{}^{\prime }=\sum_{i=1}^{x}\frac{d-d_{\text{min}}}{d_{\text{max}}-d_{\text{min}}}+\frac{\int_{1}\left(U-G\right)}{U}\in \left[0.5,1\right]. \end{array}$$

The standardization process *σ* entails converting the dataset's large and small outlier information into a random variable with an overall average value between 0 and a confidence level of 1. The subsequent (13) is utilized to perform the conversion process:

(13) $$\begin{array}{c} d{}^{\prime }=\sum_{i=1}^{x}\frac{d-{\bar{d}}_{\text{min}}}{\sigma }+d_{\text{max}}-d_{\text{min}}. \end{array}$$

Every station is composed of three layers, input nodes, hidden layers, and convolution layers, also with weight training of each layer being *β*, *γ*, and *α* including both given in the following equation:

(14) $$\begin{array}{c} \beta_{y}^{t}=\sum_{i=1}^{M}\varphi_{iy}d_{i}^{t}+\sum_{y^{\prime }}^{M}\varphi_{y^{\prime }y}q_{y^{\prime }}^{t-1}. \end{array}$$

It assumes that specific *φ*_*y*′*y*_*q*_*y*′_^*t*−1^ paper work is maintained in the RNN receptors after each cycle of data transfer. It must enter the *φ*_*y*_(*q*_*y*′_^*t*−1^) next nerve cell as new information and influence the subsequent output data which are as follows:

(15) $$\begin{array}{c} \alpha_{y^{\prime }}^{t-1}=\sum_{t⟶1}^{y}\varphi_{y}\left(q_{y^{\prime }}^{t-1}\right)+\varphi_{y^{\prime }y}q_{y^{\prime }}^{t-1}. \end{array}$$

For the respective input neurons, the original information of a hidden unit and the output variable to output units at time step *t* are as follows:

(16) $$\begin{array}{c} \gamma_{y^{\prime }}^{t-1}=\sum_{y=1}^{M}\varphi_{y0}q_{y}^{t}+\varphi_{y}\left(q_{y^{\prime }}^{t-1}\right). \end{array}$$

## 3. Results and Discussion

The resemblance of performance measures to those of algorithms as in (2); the *i*th teaching quality evaluation index is based on this to retrieve in Figure 2.

It also demonstrates that such a constructed framework performs better than conventional algorithms, including the neural network models, in trying to address activity recognition problems. Its high specificity is also confirmed by the teaching accuracy of 98.65%. The convolutional neural network might capture not only the characteristics of physiology courses based on artificial intelligence training (93.36%) and teaching (95.54%) accuracy but also loss of training (90.37%) analysis, optimise the required data, and increase the reliability of human movement recognition simply by attempting to adjust its set of parameters. The train and test graph of the neural network accuracy combined with wireless network virtual reality 5G technologies is the train and test graph of load prognostication in physiology course training using a convolutional neural network.

The *d*_*i*_*φ*_*j*_*R*_*j*_^2^ quantity of interaction optimizing parameters between the information data network and the medium surface access point is then shown in equation (6) and used in Figure 3. Also, it shows that now the trained activity recognition framework appears to provide an overall accuracy of more than 99.8%, the precision of more than 95.76%, and the recall frequency of much more than 90.82% for the different topics. Since training, the activity recognition framework for numerous physical education, the testing frame constructed convolutional neural network prototype has exceptional human activity recognition potential. Based on artificial intelligence, an activity recognition structure for various physiology courses was developed, and testing was conducted using wireless network virtual environments 5G technologies.

The isolation of the visual medium in physical training teaching, which includes higher levels of physical activity along with posture judgement, has been shown to continue providing educators with honest information about student movements, and thus, this recognition of educational physical actions can provide legitimate input to improve training performance. Although data from sophisticated wearable technology sensors were used to accurately determine human actions, structure classification remained a source of contention. The experimental results (refer Table 1) show that a convolutional network-based activity recognition system could indeed accurately recognise human behaviour with 99% accuracy. Tests for precision (90.56%), recall (89.23%), and accuracy (99.34%) were established in numerous physical education programs, followed by the human impacts of precision (90.56%), recall (84.67%), and accuracy (99.67%).

The experiment results show that the neural network's interaction weight can be defined to use the ∑_*j*=1_^*r*^*φ*_*j*_*R*_*j*_ optimization technique of a specific neural network based on Figure 4. This shows that a convolutional neural network algorithm human action recognition method combined with wireless network virtual reality 5G technologies can successfully recognise human behaviour with an accuracy of greater than 99%. It was discovered in a previous similar study that a body motion useful for detection to KNN features of regional succession instated had an 85.34 percent detection performance. The detection accuracy of an NNGA and random forest surface modification was 78.12%, surpassing the convolutional neural network GA, which had a convolutional neural network. The algorithm's efficiency is 96.34%.

It compares (refer Table 2) the analysis in different algorithms and the best performance for testing and training is provided high accuracy in CNN with AI (99%). Education in physiology courses is regarded as an important component of a reflection of the higher education teaching sector. An educator is in charge of teaching students teaching methods and/or physiology courses. This study proposed a new method of teaching analysis in physiology education classes at academic institutions. Aside from combining neural networks and algorithms, the methodology we proposed can improve the overall traditional infrastructure in terms of global consolidation and training time.

We investigated students' attitudes toward physiology education courses in online teaching, their ability to learn, and their use of educational teaching systems in this regard. Because an individual's areas of interest are roughly equivalent to ∫(*φ*_1_,…, *φ*_*x*_) ability, the description of such an optimization problem has a massive effect on genetic algorithms. Because of the close navigation companionship between the *U* − *G* optimization process and the optimization method, the *G* < *U* strength training computational methods are outlined as shown in Figure 5. A moderately sized set of questions was used to conduct an online survey from the data provided by physical education teaching. The performance analysis for impartial evaluation of school teaching specifies the mean, standard deviation, difference of mean, and difference standard error, and difference values, but it also analyses the assessment based on these values. The investigation of physical education teaching based on neural network involves determining which one is the best to represent. Physiology education courses are taught using a wireless network in 5G technology, which compares various methods of performance analysis for the median score in order to obtain the best result for the CNN with AI 5G technologies.

Despite the challenges, students think that the present face-to-face method is the best way to handle the whole teaching-learning process and that the framework should be viewed as a supplement to enable the educational process. As a result (refer Table 3), 68.32% of students prefer facial expression instruction and 62.27 percent prefer a combination of traditional and digital classes, while 17.78 percent prefer online-based instruction.

The convolutional neural network algorithm is being used to not only perform AI learning data analysis in physiology courses based on artificial intelligence combined with wireless network virtual reality 5G technologies but also extract even more important information from data besides evaluating and also modifying valuable data. It assumes that specific *φ*_*y*′*y*_*q*_*y*′_^*t*−1^ paper work is maintained in RNN receptors after each cycle of data transfer. It must enter a *φ*_*y*_(*q*_*y*′_^*t*−1^) next nerve cell as new information and influence the subsequent output data in Figure 6. Regardless of how advanced the data processing is or how much information is available, machine learning algorithms struggle to identify patterns in the data. Students stated that learning has been considered as the most important goal, so education includes guidelines, evolution, identification, knowledge, and teamwork, all of which improve student learning. The achievement of students' performance structures is dependent on behavioural quality ratings. The frequency-time(s) accuracy is based on the performance analysis, and it has been compared with various methods and represents the differences in physical education courses teaching statistics data (refer Figure 6).

## 4. Conclusions

In health education, physiology education will be perceived as a significant aspect of the educational system. The job of a physiology instructor is to provide students with instruction in physiology, with an emphasis on artificial intelligence (AI) or health. For the first time, this study used student physiology courses to examine teacher quality in higher education courses. Combining neural network algorithms with wireless network methods in the framework proposed by humans could indeed improve the general broad validity of conventional wireless networks and training time. As a reflection of 5G's virtual reality capabilities, health education is seen as a key component of the system. This study used student physiology classes to develop a novel approach to assessing instructor quality in higher education courses. Conventional wireless networks can be used more widely with less training time if the framework proposed by humans is combined with neural network algorithms. The study proved that CNN with AI technique has obtained accuracy of 99%. It states that the proposed algorithm works well than the existing algorithms.

## Figures and Tables

**Figure 1:** Proposed model for the physiology course.

**Figure 2:** The neural network training and testing graph physiology courses based on artificial intelligence combined with wireless network virtual reality technology in the context of 5G.

**Figure 3:** The result analysis for human activity recognition framework for various physiology courses based on artificial intelligence: the testing set with wireless network virtual reality 5G technologies.

**Figure 4:** The physical educational courses in human activity recognition accuracy using a CNN algorithm with wireless network virtual reality 5G technologies.

**Figure 5:** Performance analysis physiology courses: median scores and differences in physical education teaching statistics with wireless network in 5G technology.

**Figure 6:** Comparison and performance analysis training load prediction in physiology education courses, teaching based on convolutional neural network statistics.

**Table 1:** Result analysis for various physiology courses based on artificial intelligence: the testing set with wireless network virtual reality 5G technologies.

Technology implementation	Precision(%)	Recall(%)	Accuracy(%)
Various physiology courses	0.90	0.88	0.98
Human activity wireless network virtual reality 5G technologies	0.93	0.82	0.99

**Table 2:** Comparison analysis for various algorithms.

Algorithm	Training	Testing	Accuracy
NNGA	0.79	0.73	0.75
KNN	0.83	0.89	0.83
Random forest	0.78	0.83	0.79
CNN with AI	0.99	0.98	0.99

**Table 3:** Impartial measurements test of physiology education courses, teaching load prediction on convolutional neural network.

Parameters	Mean	S. D.	Meandifference	Std. errordifference
The online environment	4.24	2.37	−0.46	0.26
Online-based teaching	3.26	2.54	−0.53	0.26
Platform use	3.87	3.82	0.08	0.43
Platform usefulness	3.93	3.28	−0.41	0.42

## Data Availability

The data used to support the ﬁndings of this study are available from the corresponding author upon request.
